The article "Pancreatic Cancer Survival Prediction: A Survey of the State-of-the-Art" was published in 2021. Journal: Comput Math Methods Med.

# Pancreatic Cancer Survival Prediction: A Survey of the State-of-the-Art

**DOI:** 10.1155/2021/1188414

**Published:** 2021-09-30

**Authors:** Wilson Bakasa, Serestina Viriri

**Affiliations:** School of Mathematics, Statistics and Computer Science, University of KwaZulu-Natal, Durban, South Africa

## Abstract

Cancer early detection increases the chances of survival. Some cancer types, like pancreatic cancer, are challenging to diagnose or detect early, and the stages have a fast progression rate. This paper presents the state-of-the-art techniques used in cancer survival prediction, suggesting how these techniques can be implemented in predicting the overall survival of pancreatic ductal adenocarcinoma cancer (pdac) patients. Because of bewildering and high volumes of data, the recent studies highlight the importance of machine learning (ML) algorithms like support vector machines and convolutional neural networks. Studies predict pancreatic ductal adenocarcinoma cancer (pdac) survival is within the limits of 41.7% at one year, 8.7% at three years, and 1.9% at five years. There is no significant correlation found between the disease stages and the overall survival rate. The implementation of ML algorithms can improve our understanding of cancer progression. ML methods need an appropriate level of validation to be considered in everyday clinical practice. The objective of these techniques is to perform classification, prediction, and estimation. Accurate predictions give pathologists information on the patient's state, surgical treatment to be done, optimal use of resources, individualized therapy, drugs to prescribe, and better patient management.

## 1. Introduction

Radiologists detect pdac tumours by symptoms of the disease and patient history but not image processing. This paper studies some ML techniques used in image processing to predict pdac overall survival. The anatomy of the pancreas is shown in Figure 1.

Cancer on the pancreas is a challenge because it is difficult to detect. As there are no clear signs in the early stages, it metastasises rapidly, having a poor forecast of the future course of the disease. The early stages of the diseases show no symptoms. In the later stage, the patient will have a lack of appetite and weight loss.

Medical experts recommend knowing the tumour type as each has a different treatment and behaves in different ways. Researchers estimated that 94% of exocrine tumour patients suffer from pdac type [3].  Figure 2 shows a pdac [4]. Tumour size has a significant influence on overall survival rates. A larger tumour is difficult to treat through resection.

Accurate predictions are crucial as they give pathologists information on state of the patient, surgical treatment to be done, optimal use of resources, provision of individualized treatment, drugs to prescribe, and better management of the patient. Features used for prediction include genomics and proteomic data, clinical factors, and pathological images. The need to identify possible weaknesses including experimental design, data collection from valid sources, and the analysis and result validation is a vital step as it affects the prediction of clinical decisions [5, 6].

ML techniques classify pdac patients and learn to predict the best survival period for each patient. Classify pdac stages into low, medium, or high-risk groups. ML techniques have been used to model the progression and treatment of pdac conditions. ML tools are powerful in identifying features from large datasets, which makes them of great use [7].

Big data with the increased patient will stress doctors, making them more error-prone when making critical decisions concerning human life. Machines can manage these large sets of imaging data with a lower error rate, attested by the unfitness of medical personnel to colligate and see the big picture from imaging data. Machines can help them by assessing large numbers of image datasets and determine whether there are any patterns suspicious to be cancerous. Machines also can assist by superseding doctors or specialist at times of their absence and provide the diagnosis in even critical cases [8].

Predictive technique models such as ML (statistical multivariate regression and deep learning (DL)) can be used for pdac survival rate prognosis. The techniques have to be reinforced for best predictive performance.  Figure 3 shows the steps to follow during the prediction process. This paper will compare imaging techniques used in the medical world, including magnetic resolution imaging (MRI) and computed tomography (CT). These imaging techniques produce images that need to be segmented into pixel classes. In a review of segmentation methods, including those used in deep learning, the current technology is mostly used in overall survival prediction for pancreatic cancer patients. The feature extraction techniques are then looked at, leading to classification after the necessary features to be extracted. Deep learning techniques implemented in feature extraction and classification are then summarised.

## 2. Medical Imaging Techniques

Medical imaging is a technique and process used to look at the human body, diagnose, monitor, or treat medical statuses, including a visual representation of the functions done by some organs or tissues. Imaging techniques help screen for hidden features before visible symptoms, diagnose the conditions that would have developed into the now visible symptoms, and manage the disease stages or reaction to possible treatment. This help to predict the overall survival of pdac patients. Common imaging techniques are computed tomography (CT) scan and magnetic resonance imaging (MRI).

Blood and other laboratory tests usually determine the existence of pdac. In imaging the pancreas (Figure 4), computed tomography (CT) and magnetic resonance imaging (MRI) were used to help determine if the condition exists. If detected, then determine the stages and reaction to treatment, making it possible to predict the patient's overall survival rate.

## 3. Segmentation

Segmentation is an image processing proficiency for bisecting an image into multiple regions. The process of segmentation well define semantic entity boundaries in an image, as shown in Figure 5. Pixel in the image is allocated labels to match affiliation according to their semantic properties.

Segmentation can be defined as a map of the greyscale into the binary set {0, 1}.

(1) $$\begin{array}{c} s\left(x,y\right)=\left\{\begin{array}{c} 0\text{ if }g\left(x,y\right)<T\left(x,y\right),\\ 1\text{ if }g\left(x,y\right)\geq T\left(x,y\right). \end{array}\right. \end{array}$$

Images are segmented using a graph cut with some cost, formed from image pixels. Image pixels of similarity and nearby are put in the same zone [13, 14]. Graph cut *T* cost (where *T* is a set of edges) is the sum of the edge weights of the cuts.

(2) $$\begin{array}{c} X_{\text{cut}}=\underset{\left(i,j\in T\right)Z_{ij}}{\sum }\;, \end{array}$$

where *Z*_*ij*_ represent edge weight *i*, *j* from node *i* to node *j* in the graph and cut and *T* represents all the edges' sum. In graph cut segmentation, a graph image section is zoned such that the cut cost *X*_cut_ is reduced.

Segmentation of an image *M*_*o*_ is a pair (*∂Ω*; *M*), where *M* is some approximation of *M*_*o*_, where *M*_*o*_ is defined in *Ω*. The energy associated with a segmentation (*∂Ω*; *M*) is the sum of three terms:

(3) $$\begin{array}{c} Z\left(\partial \Omega ,M\right)=\alpha \mathrm{int}\left(\frac{\Omega }{\partial \Omega }{\left|\nabla M\right|}^{2}dx+\beta \text{length}\left(\partial \Omega \right)\right.+\mathrm{int}\left(\frac{\Omega }{\partial \Omega }\left.{\left(M-M_{o}\right)}^{2}dx\right).\right. \end{array}$$

If *M* is imposed to be constant within each region,

(4) $$\begin{array}{c} Z\left(\partial \Omega ,M\right)=\alpha \text{length}\left(\partial \Omega \right)+\mathrm{int}\left(\frac{\Omega }{\partial \Omega }{\left(M-M_{o}\right)}^{2}dx\right). \end{array}$$

Gradient operator and Laplacian operator are defined as follows:

1. *Gradient Operators*. The gradient of an image, *f*(*x*; *y*), at a location (*x*; *y*) is defined as the vector.

(5) $$\begin{array}{c} \nabla f\left(x,y\right)=\left(\begin{array}{c} g_{x}\\ g_{y} \end{array}\right)=\left(\begin{array}{c} \frac{\partial t}{\partial x}\\ \frac{\partial t}{\partial y} \end{array}\right). \end{array}$$

(2) *Laplacian Operator*. The Laplacian of an image *f*(*x* : *y*) is defined as follows:

(6) $$\begin{array}{c} \nabla^{2}f\left(x,y\right)=\frac{\partial^{2}f\left(x,y\right)}{\partial x^{2}}+\frac{\partial^{2}f\left(x,y\right)}{\partial y^{2}}. \end{array}$$

Medical images from CT and MRI modalities require segmentation to fix various abnormalities like tumours and cancerous elements. Most methods that use feature-based approaches currently rely on the attributes of features extracted by a human specialist. This poses some challenges as humans are prone to making errors and miss potential features for the segmentation of the image. DL addresses the issue by providing automated feature learning techniques. The mostly used technique in computer vision is convolutional networks [15, 16]. The other used algorithms in computer vision include generative adversarial networks (GNAs), and variational autoencoders (VAEs) are used to solve challenges like the generation of images. The scale-invariant feature transformation (SIFT) is another object detection algorithm used for tumour detection within images regardless of the image rotation, orientation, or scale [17].

Texture features can be used according to [18] and implemented with other methods like the Bacterial Foraging Algorithm (BFA) used for classification. Studies have shown that CAD system, Haar wavelet transform, and clustering methods can be implemented for accurate diagnosis and processing of pdac images obtained from MRI and CT modalities, as shown in Table 1.

Different images call for different segmentation techniques as they have distinct feature and properties as envisioned in terms of colour (greyscale images, binary images, and colour images) and texture (texture images and nontextured images) [23].  Table 2 shows the advantages and disadvantages of some different segmentation techniques used.

## 4. Segmentation Using Deep Learning Techniques

Segmentation techniques continue to be developed and improved to solve challenges differently. The evolution of convolutional neural networks has seen most techniques developed, as shown in Tables 3 and 4. Based on architecture or framework, these techniques are grouped into an instance or semantic segmentation [30].

In the semantic segmentation process, a label is assigned to every pixel in the image, which is different from classification, assigning a single label to the entire picture. Semantic segmentation treats multiple objects of the same class as a single entity and involves detecting objects within an image and grouping them based on defined categories.

In the instance segmentation process, multiple objects of the same class are treated as distinct individual objects or instances. It involves detecting objects within defined categories, and it is more complicated than semantic segmentation.

### 4.1. GoogLeNet [31]

CNN layers are stacked as networks in networks, based on the concept of [32]. GoogLeNet is built from many inception modules of various filter sizes applied to the input and the concatenated outputs. These inception modules and filters are contained within the stem, a standard architecture that simultaneously provides the extraction of image features at varying levels of detail. GoogLeNet does not use fully connected layers, instead uses global average pooling, thus lessening model parameters required.

### 4.2. ResNet [31]

Train much deeper networks making use of skip connections. The authors trained a 152-layer deep ResNet, and they also successfully trained a version with 1001 layers. Combining the power of skip connections in addition to the standard pathway allows the network to copy activations from every ResNet block or layer, maintaining information during processing through layers. Various features are finest assembled in external networks, as some need extra depth. The skip connections facilitate both simultaneously, improving the network's flexibility when given input data. Skip connections allow the network to learn residuals, thereby giving ResNets an advantage to perform a boosting.

### 4.3. U-Net [33, 34]

U-Net is a very popular and successful network for segmentation in 2D images. When fed an input image, it is first downsampled through a “traditional” CNN before being upsampled using transpose convolutions until it reaches its original size. In addition, based on the ideas of ResNet, there are skip connections that concatenate features from the downsampling to the upsampling paths. It is a fully convolutional network, using the concepts first introduced in [35].

### 4.4. V-Net [34]

V-Net is a three-dimensional version of U-Net with volumetric convolutions and skip connections as in ResNet.

## 5. Feature Extraction Techniques

A technique of transmutation to exhume common characteristics and shape in an image, extracting the image properties that differentiate it from a range of images. CT and MRI images are complicated, and methods of feature extraction application on them are limited. Image features can be considered the fundamental attributes or prominent features for realizing the image. As in Table 5, feature extraction methods use four image features, texture features, colour image features, shape features, and spatial relations [46–48]. In [49], the author classified feature extraction into topological and geometric features, statistical features, and series expansion features and global transformation.

Many researchers have studied the detection of skin cancer, breast cancer, and brain cancer. Different algorithms have been successfully applied for the early diagnosis of these tumours. Artificial neural networks (ANNs) have been implemented for detecting skin cancer [50]. They preprocessed the image to remove noise and enhance the image. The wavelet transform was used for feature extraction, and then, the tumour was classified using backpropagation neural networks.

The features must depict the objects correctly for classification. Shape features and feature extraction methods can both be based on either boundary characteristics or regional characteristics. The methods of shape feature extraction are boundary-based and region-based. Shape feature extraction lacks a mathematical model, and if changed, the result is not reliable, and accuracy depends on the presegmentation effects [49, 51–55].

Wavelet decomposition is used for brain tumour detection. The grey-level cooccurrence matrix (GLCM) is used for feature extraction, while probabilistic neural networks are used for further classification [56]. Another algorithm for brain tumour detection is using an artificial neural network fuzzy inference system [57]. Various supervised learning techniques are used to detect breast cancer. These include principal component analysis (PCA) for feature extraction and support vector machines (SVMs) and k-nearest neighbour for classification [5]. As seen above, the various parametric and nonparametric classifiers can be used to classify and detect different tumours based on the tumour's features.

Dimension reduction is used in machine learning and statistics to reduce the number of feature set, categorized into feature selection and feature extraction [58, 59]. Feature extraction is referred to as dimensionality reduction [60]. The input matrix *W*, of dimension *A* × *B*, is

(7) $$\begin{array}{c} \left[\begin{array}{ccc} W_{11} & \cdots & W_{1B}\\ \vdots & W & \vdots \\ W_{A1} & \cdots & W_{AB} \end{array}\right], \end{array}$$

where we have a sample representation by rows and variables represented by columns. The feature extraction algorithm will learn from this transformation the prerequisite features needed for extraction.

Image texture analysis is currently used to predict tumour heterogeneity. However, only a few studies have reported texture analyses of tumour heterogeneity in pdac [61].

Edge detection highlights the contrast or difference in the intensity of an image. This detection draws attention to the boundaries of features within an image, the same way a human vision can perceive the perimeter of an object, which is of different contrast to its environment. Fundamentally it is the boundary of an image that varies in intensity levels or the contrast [13, 14, 62]. The edge is at the location of the variation and is detected by differentiation of first order. Intensity variation is demonstrated by varying adjacent pixels. If computed on image *M*, the horizontal detector edge creates an intensity variation between two horizontally adjacent points, as such detecting the vertical edges, VE(*x*), as follows:

(8) $$\begin{array}{c} \text{V}{\text{E}}_{X_{xy}}=\left|M_{xy}-M_{x+1,y}\right|\forall x\in 1,N-1;y\in 1,N. \end{array}$$

A vertical edge detector that varies adjacent vertical points is needed to detect horizontal edge using vertical edge detectors, VE(*y*), as follows:

(9) $$\begin{array}{c} \text{V}{\text{E}}_{X_{xy}}=\left|M_{xy}-M_{x,y+1}\right|\forall x\in 1,N;y\in 1,N-1. \end{array}$$

We can then combine the two forming an operator VE(*y*) that detect both vertical and horizontal edges. That is,

(10) $$\begin{array}{c} \text{V}{\text{E}}_{X_{xy}}=\left|M_{xy}-M_{x+1,y}+M_{xy}-M_{x,y+1}\right|\forall x,y\in 1,N-1, \end{array}$$

which gives

(11) $$\begin{array}{c} \text{V}{\text{E}}_{X_{xy}}=\left|2\times M_{xy}-M_{x+1,y}-M_{x,y+1}\right|\forall x,y\in 1,N-1, \end{array}$$

given the coefficients of a varying template which can be twisted together with an image to detect all the edge points.

Grey-level cooccurrence matrix (GLCM) and histogram analyses are methods employed by texture analyses to classify objects according to their texture. Evaluation of grey level placement, regularity, and coarseness within the damaged or abnormal change in the pancreatic tissues, computer vision, and machine learning algorithms can analyze CT and MRI images to provide other morphological details related to pdac tumour heterogeneity.

## 6. Survival Prediction Model Review

Traditional diagnosis models like the popular American Joint Committee on Cancer (AJCC) tumour-node-metastasis (TNM) model is used in cancer diagnosis. According to [7, 8], the challenge is that they do not predict the cancer patient's overall survival. The study explores different ML techniques used in pdac survival rate prediction.

ML techniques classify pdac patients and learn to predict the best survival period for each patient. Classify pdac stages into low, medium, or high-risk groups. ML techniques have been used to model the progression and treatment of pdac conditions. ML tools are powerful in identifying features from large datasets, which makes them of great use.

Big data with the increased patient will stress doctors, making them more error-prone when making critical decisions concerning human life. Machines can manage these large sets of imaging data with a lower error rate, attested by the unfitness of medical personnel to colligate and see the big picture from imaging data. Machines can help them by assessing large numbers of image datasets and determine whether there are any patterns suspicious to be cancerous. Machines also can assist by superseding doctors or specialist at times of their absence and provide the diagnosis in even critical cases. ML can be either supervised learning or unsupervised learning, as shown in Figure 6.

Supervised learning (Figure 7) is typically implemented in the context of classification, mapping the input to output labels, or regression, for the mapping of input to continuous output.

For both regression and classification, the goal is to find specific relationships or structure in the input clinical data for the correct generation of output patient clinical data, determined entirely from the clinical training data. When carrying on supervised learning, the principal circumstances are model complexness and the bias-variance tradeoff.

Model complexity refers to the complexness of the function sought to learn.  Figure 8 shows the data analytics types, indicating the complexity of each type. The proper level of model complexity is determined by the nature of patients' clinical training data, the smallness of data, and distribution throughout different possible assumptions.

Unsupervised learning requires representation learning, density estimation, and clustering to be carried out. We need the inherent structure of our patients' clinical data without using explicitly provided labels. Since no labels are provided, there is no specific way to compare model performance in most unsupervised learning methods. Exploratory analysis and dimensionality reduction are the common use cases for unsupervised learning. Unsupervised learning is powerful for the identification of hidden structures in patients' clinical data. Over the years, survival prediction models in cancer were developed implementing techniques like Decision Trees (DTs), support vector machines (SVMs), Bayesian Networks, and artificial neural networks (ANNs). There is a need to validate these machine learning methods used in progression analysis of cancer for them to be used in medical practices.

ML has been implemented in cancer prognosis or overall survival prediction [63]. Most of the studies proposed for the last years focused on developing predictive models using supervised ML methods to predict disease outcomes [64] accurately. Based on the analysis of their results, it can be concluded that the integration of multidimensional heterogeneous data, with the application of different models for feature selection and patients' data classification, can help to model useful tools for overall survival prediction for pdac patients [65].

Many evolutionary algorithms have been implemented into resolving challenges to do with feature selection and classification to analyze gene expression data. Genetic algorithms [65–67] are implemented for creating selectors with each allele is linked to one gene and having a state to tell if selected or not. Genetic programming is practically applicable to find hidden features in complex datasets. It is good for identifying rule-based classifiers and gene expression profiling from medical data.

A random survival forests method for the analysis of right-censored survival data was suggested by [68]. New survival splitting rules for growing survival trees and a conservation-of-event principle for survival forests are proposed to define an interpretable measure of mortality used as a predicted outcome.

Some papers proposed the use of Feed Forward Neural Networks. ANNs [69] were implemented for two years on patients and the network predictions for twelve months of death compared to surgical doctors. ANNs achieved a 95% prediction accuracy [32].

The techniques can detect features from complex datasets. According to [66], genetic programming can make an automatic feature selection. They showed that genetic programming performs substantively better than SVM, multilayered perceptron, and random forests in classifying. As reported by [70], the result indicated frequency usage of ANN with high accuracy in survival prediction of any malignancy. However, they suggested combining ANN and fuzzy logic with 93% accuracy as superior and powerful.

A short review of current algorithms being used in ML such as SVM [71–73], Naïve Bayes [74], Logistic Regression [75], genetic algorithms, Decision Tree, ANN, and KNN algorithm is done. A graph-based semisupervised learning paradigm that takes advantage of both unlabelled and labelled data when training a model is used. Other semisupervised learning (SSL) are self-training, cotraining, and transductive SVM.

According to the study [76], for lung cancer, the study chooses Linear Regression, Decision Trees, Ensemble Learning algorithm, random forest, and Gradient Boosting Machines as logistic-based methods. SVM was then used to sum the predictions of each of the five models into final predictions. The study by [77] concluded that classification and regression trees (CARTs) are also used compared to ANN as prediction modes. ANN proves significantly more accurate than the CART model. The comparison of three different techniques is in [78], SVM, Decision Trees, and k-nearest neighbour. SVM proved to be the best performer.

However, in [79], the extracted features are used as inputs for Back Propagation NN and Logistic Regression (LR) and the two algorithms are compared for accuracy. LR was the best given a higher number of features. Random forest [80] was used as a biomedical classifier that has led to the proposal of two variants, namely, Forest-RK and dynamic random forests [81].

In survival prediction for cancer [35, 82–84], they used convolutional neural networks (CNNs) for classification and feature extraction with the aid of computer-aided diagnosis (CAD) based on pathological images. Tumours can be characterized through the implementation of supervised ML [85] for labelled data, and usage of SVM as state-of-the-art classification algorithms. Experiments to prove state-of-the-art ML techniques can be efficiently or equally better than traditional techniques (Linear and Logistic Regression) were done [86]. All algorithms executed using Weka ML workbench. ML algorithms used are Linear Regression, ZeroR, and Logistic Regression. For classification, the algorithms they used are Naive Bayes, J4.8 (C4.5 learning algorithm), k-nearest neighbor, OneR, Locally Weighted Learning, and Bayesian Nets.

Colon cancer predictions [87] implemented a supervised classification technique. Synthetic Minority Oversampling Technique (SMOTE) was used to balance the survival and nonsurvival classes. Ensemble Voting of three classifiers was found to result in the best prediction performance in prediction accuracy and area under the receiver operating characteristic (ROC) curve. The study by [88] proposed a semisupervised model in trying to address data scarcity in cancer datasets. Ensemble classifiers used to learn unlabelled data. CART tools helped to deal with missing attribute values by using the surrogate splitting technique. ML techniques can be categorized into the following:

1. Statistical techniques
2. Deep learning (DL)

### 6.1. Statistical Techniques

According to [3, 63], Weibull distribution is implemented to estimate the overall survival. It is the widely used technique for statistical cases involving data with periods, which considers life behaviour. The author states that alpha is the rendering probability of 63.2% prediction that an event occurs. Beta is used to represent the probability of growing (beta > 1) and to decrease (beta < 1). If nearing one, then the distribution is exponential with an invariable chance rate.

The study [8, 89] used the cox proportional hazard to assess the independent effects of prognosis factors. It was also implemented to assess the correlation between tumour node metastases (TNMs) [63]. Song et al. [8] used a Student's *t*-test or chi-square test to compare disease features. The Kaplan-Meier was used for the assessment of survival factors. The rank test was used to test survival curve variation. They argued that their model is capable of providing quantitative prognosis to individual cancer patients. Song et al. and Hang et al. [8, 89] designed a graphical nomogram using the R statistical package using statistical analysis. The c-index was applied to validate the predictive accuracy of the nomogram.

### 6.2. Deep Learning

Deep learning is a subset of ML, in which algorithms learn unsupervised from unstructured or unlabelled data. Deep neural networks (Figure 9) are designed based on biological neural networks with many hidden layers to extract features from data using interconnected node matrix to imitate how the human brain works.

A node is the basic unit of an artificial neural network. The input feature set is multiplied by corresponding weights using mathematical functions, passing the output to the next node layer. These outputs are weighed up to known facts. It autoadjusts the weights using errors as feedback to minimise future errors during iterations [90, 91].

Deep learning rose to its prominent position in computer vision when neural networks started outperforming other methods on several high-profile image analysis benchmarks.

The main common characteristic of deep learning methods is their focus on feature learning: automatically learning data representations. Discovering features and performing a task are merged into one problem and therefore both improved during the same training process [31].

Tumour detection in pancreas images is achieved using CNN, which extracts the image features, classifying the tumour based on the extracted features. Various classifiers used for feature extraction in machine learning include Naive Bayes classification, support vector machine, and logistics functions. CNN delivers the information needed using convolution methods in three steps: convolution, pooling, and padding, which are layers in the input and output images. Region Convolution Neural Network (R-CNN) is used to extract image features from a particular region. The CNN will be acting as a feature extractor.

[92] suggested deep learning and described it as in the unsupervised learning category. Segmentation using CNN is mainly used for image processing in machine learning. It requires providing segments of the pancreas image to the convolution neural network as the inputs. CNN labels the pixel and classifies each pixel determining the context to identify the images. A segment represents the tumours in the pancreas image or parts or the superpixels. Analysis of the images is carried out in three levels: classification, tumour detection, and segmentation. Segmentation significantly detects the tumour, classifying them into their different classes.

#### 6.2.1. Deep Learning Frameworks and Image Processing Platforms

Developing complex machine learning models for image processing requires special platforms and frameworks. Some of the popular frameworks are TensorFlow and PyTorch.

*(1) TensorFlow [93]*. Google developed TensorFlow, which is an open-source framework with support for machine learning and deep learning. TensorFlow facilitates the creation and training of custom deep learning models. The framework has a set of libraries, including for image processing projects and computer vision applications.

*(2) PyTorch [94]*. PyTorch is an open-source deep learning framework designed by the Facebook AI Research lab (FAIR). This Torch-based framework has Python, C++, and Java interfaces. PyTorch is used for building computer vision and image processing applications.

#### 6.2.2. Neural Networks in Image Processing

Researching on neural networks has been done for many years, which has seen improvements in machine learning, a reason for the magnificent progress in medical imaging and computer vision technology today. Most successful machine learning models for image processing implement neural networks and deep learning. Examples include Mask R-CNN and fully convolutional networks.

*(1) Mask R-CNN*. Mask R-CNN [95] is a Faster R-CNN-based deep neural network that separates tumours in a processed image. This neural network performs segmentation and generates masks and bounding boxes. The neural network is adjustable, flexible, and efficient as compared to other techniques. Mask R-CNN is poor in real-time processing, as the neural network is massive and the mask layers slow performance, mainly if compared to Faster R-CNN. For instance, segmentation, Mask R-CNN is a very efficient technique.

*(2) Fully Convolutional Network (FCN)*. FCN [40] was developed by University of Berkeley researchers. CNN has a convolutional layer rather than FCN, which has a regular, fully connected layer. This difference enables FCN to manage various input sizes. Also, FCNs use downsampling and upsampling to reduce computational costs for convolution functions.

## 7. pdac Survival Prediction

There is a possibility that delay in diagnosing pdac can cause concentrated resectable tumours to develop into unresectable by the time of diagnosis [96]. They estimated that it might take just over one year for an average T1-stage pdac to develop into a T4-stage tumour. CT/MRI scans taken by radiologists for other medical purposes but not focused on the pancreas are useful for screening pdac at a reduced cost, time, or radiation exposure [97]. Deep learning has proven to serve as a tool at the disposal of a radiologist in computer-aided diagnosis that points to minor changes on the pancreas that may result in abnormalities that health experts could miss.

A few studies have evaluated the detection of pdac tumours using deep learning techniques [98]. According to [99], they study CT scans using deep learning networks from 303 pdac patients and 136 normal test data. The results showed the detection of pdac had 94.1% sensitivity and 98.5% specificity. The study by [100] used 370 patient CT scans suffering from pdac and 320 test data to study the effectiveness of deep networks in pdac tumour detection. A 98.8% accuracy, 99.3% specificity, and 98.3% sensitivity were achieved. The study proved that a deep network, if implemented in detecting pdac, is more sensitive than radiologists. The results indicated that about 91.7% of tumours missed by radiologists could be correctly classified by deep network and paying attention to tumours less than 2 cm in size, achieving a 92.1% sensitivity.

The advantage is that deep learning has over traditional methods, as the networks can adapt automatically and modernise features from big data instead of already added features. Deep learning is effective in that it can receive new complex pancreas image feature representation quickly [92].

Convolutional neural networks (CNNs) are a category of deep learning networks developed precisely for image processing. The networks have neurons that mimic neurons in the human brain. CNNs need fewer preprocessing operations than other neuron networks, and the networks learn the required filters and characteristics during training rather than using hand-engineered filters. They are multilayered neural networks with layers organised in three dimensions: weight, height, and depth. They have two components: feature extraction and classification [17, 98, 100].

Fully convolutional network (FCN) is suitably implemented in image segmentation tasks when the neural network splits the processed image into many pixels to be labelled and classified. Popular examples of FCNs for semantic segmentation are RefineNet and DeepLab.

U-Net is a convolutional neural network that allows for fast and precise image segmentation. U-Net was designed particularly for the segmentation of complex tasks in biomedical image processing. U-Net is built with U-shaped architecture with more feature channels in its upsampling part so that the network propagates context information to higher-resolution layers [34].

In feature extraction, CNN runs many convolutions and pooling functions to detect features used for image classification. The network algorithm predicts the tumour in the pancreas image with a calculated probability in the classification component.

Techniques employing deep learning are used in the prediction and prognosis of pdac development. They focus on three major domains: prediction of cancer susceptibility, prediction of pdac relapse, and prediction of pdac survival rate. This paper focuses on the third case, which predicts several possible parameters characterizing pdac development like survival time, life expectancy, and progression. The overall survival rate and the pdac relapse mostly depend on the medical treatment and the quality of the diagnosis [101].

## 8. Dataset

According to the study [102], they used the Cancer Imaging Archive (TCIA) Public Access dataset, consists of 3D CT scans of 512 × 512-pixel resolution from 53 males and 27 female subjects of the 18-76 age group. Liu et al. [100] implemented CNN to the Taiwanese Centre dataset with contrast-enhanced CT images of 370 patients with pdac and 320 controls. These datasets can be used to study the prediction of pdac overall survival using CT images and ML or deep learning techniques.

## 9. Period for Prediction

According to [63], they considered one year, three years, and five years, but [87] reduced the three years to two. While in [65], high or low was used. Follow up for five years [32] and predict death within nine, twelve, fifteen, eighteen, twenty-one, and twenty-four months. However, they differ with [7] as they used six, twelve, and twenty-four months. Short periods of survival times like less than six months give better accurate results when developing a prediction model [103]. Some authors [89] used three risk groups with median overall survival of 11.7, 7.0, and 3.7 months. Short- and long-term classes were used by [104, 105]. According to [77], five-year survival was output prediction with zero for dead and one for alive and classified as good, intermediate, or poor.

## 10. Validation Methods

In the study of Kourou et al. [65], the methods used for evaluating the performance of a classifier are the holdout method, bootstrap, random sampling, and cross-validation. According to [8, 89], they validated their nomogram using discrimination and calibration and using bootstrap resampling. Discrimination between survival probability and actual observation was evaluated using c-index. Calibration plot was constructed to determine the concordance of predicted survival and actual survival.

Tenfold cross-validation methods were employed [76] to measure the unbiased estimate of the prediction models (DTs, ANN, and SVM). Nevertheless, [104] called it *k*-fold cross-validation, depending on the factor (*k*) used. According to [105], they used a leave-one-out-cross-validation (LOOCV) protocol.

## 11. Conclusion

This paper reviews machine learning techniques implemented in overall survival prediction of pancreatic cancer patients, that is, statistical and DL methods. ML methods have significantly proved to be effective if applied to the overall survival prediction of pdac. Features used for prediction include genomics and proteomic data, clinical factors, and pathological images. The need to identify possible weaknesses in experimental design, data collection from good sources, and the analysis and validation results is vital as it affects the prediction of clinical decisions. There is a need for a model that could help in the individualized survival prediction calculation and provide specific treatment decisions. Based on the reviews done on most studies, we have found that for the integration of various feature extraction, segmentation, and classification, DL techniques can provide a useful prediction tool best to make accurate predictions that will assist pathologists in making informed decisions.

Implementing frameworks and platforms like PyTorch and TensorFlow in developing computer vision and image processing significantly improves the overall survival prediction for pdac patients. Various neural networks are deployed to solve various image processing tasks, from binary classification to instance segmentation. Selecting the proper type and architecture of a neural network is important in creating an efficient machine learning-based image processing solution. The most used neural networks in DL are CNN and FCN. The U-Net model is largely implemented in image processing tasks and has shown a high degree of accuracy.

The authors suggest reinforcing different DL techniques in order to come up with an efficient pdac predictive model. An end-to-end model that will use DL techniques to predict the overall survival rate of pdac patients is proposed.

## Figures and Tables

**Figure 1:** Pancreas [1]. Pancreatic cancer tumours are of two types [2], exocrine and endocrine tumours. The position of origination determines this. The pdac originates from the lining of the ducts in the pancreas.

**Figure 2:** Pancreatic cancer tumour [4].

**Figure 3:** Prediction model process—started by identifying the problem and collecting related data, cleaning, and processing. The output data is passed as input through DL techniques, and a prediction is made.

**Figure 4:** Medical imaging techniques [9–12]: images from CT and MRI modalities.

**Figure 5:** Image bisection [13, 14].

**Figure 6:** Types of machine learning: supervised learning, unsupervised learning, and reinforcement learning (a hybrid of supervised and unsupervised learning).

**Figure 7:** Supervised machine learning: accept training data in labelled test data (CT and MRI images). The trained ML algorithm output plus new data is taken into the predictive model to make pdac patients' survival prediction.

**Figure 8:** Data analytics types: four types of data analytics—descriptive analysis (problem definition), diagnostic analysis (identify cause), predictive analysis (outcome forecasting), and prescriptive analysis (rules).

**Figure 9:** A deep neural network basic illustration. New data features (input layer (*i*)) are examined by many interconnected nodes (hidden layers (*h*)) that form the hidden layer generating the output (output layer (*o*)). The weights are represented by *w* where *n* = 4.

**Table 1:** pdac tumour segmentation algorithms in medical imaging.

Study	Medical modality	Proposed segmentation method	Results
Tam et al. [19]	CT	Region growing algorithm	Efficient: Jaccard index of 73.37–86.97
Balakrishna et al. [20]	CT	MATLAB	Detecting edges, corners, and points differentiating images
Sindhu et al. [18]	MRI	Texture extraction with BFA	Texture feature extraction with BFA has an accuracy of 89%.
Farag et al. [21]	CT	Cascaded superpixel segmentation	Superpixels preserve more boundaries. Dice coefficient of 70.7% and Jaccard index of 57.9%
Reddy et al. [22]	MRI and CT	K-means clustering and Haar wavelet transform	Based on threshold value with a mean threshold of 8.88

**Table 2:** Advantages and disadvantages of different segmentation techniques.

Segmentation technique	Advantage	Disadvantage
Region-based [16, 23, 24]	(i) High speed of operation (ii) Efficient for object and background with high contrast (iii) Easier to classify and implement (iv) Best when easy to define region similarities (v) Less sensitive to noise compared to edge detection	(i) Poor segments if there is low greyscale (ii) Are by nature sequential and quite expensive both in computational time and memory (iii) Region growing has inherent dependence on the selection of seed region and the order in which pixels and regions are examined

Fuzzy theory-based [25–27]	(i) The single fuzzy rule applied to stress the importance attached to feature-based and spatial information in the image (ii) Structure of the membership functions and associated parameters automatically derived	(i) Sensitive to noise (ii) Computationally expensive (iii) The determination of fuzzy membership is not very easy

Artificial network-based [15]	(i) Simple programming (ii) Make use of neural net parallelism	(i) Long training time (ii) Initialization could influence the outcome

Generalized PCA (principle component analysis) [28, 29]	(i) Low noise sensitivity (ii) Lack of redundancy of data (iii) Increased efficiency (iv) Reduced overfitting	(i) Independent variables become less interpretable (ii) Data standardization is a must before PCA (iii) Information loss

**Table 3:** Segmentation techniques: dice coefficient (DC), image dimension (ID), application (App), reference (Ref), convolutional neural network- (CNN-) conditional random field (CRF), named entity recognition (NER), maximum entropy Markov models (MEMM), and hidden Markov model (HMM).

Method	Advantages	Disadvantages	Dataset	DC	ID	Modality	App	Ref
CNN-CRF [36, 37]	(i) Flexible enough in terms of feature selection (ii) Better for NER than MEMM and HMM	(i) High computational complexity of the algorithm training stage algorithm (ii) Difficulty in retraining the model when new training data is available	Data in hospitals	86.0	2D	MRI	Brain tumour	Feng et al.

U-Net [33, 38]	(i) Provides pixel-accurate semantic segmentation (ii) It is fast to compute (iii) Its architecture is easy to understand	(i) Significant memory requirement as lower level features have to be stored for further concatenation in the upsampling phase	1245 CT images	73.6	3D	CT	Pulmonary nodules	Tong et al., Du et al.

E-Net [39]	(i) Significantly faster (ii) Provides a high frame rate for real-time applications (iii) Small storage requirements alleviating the need for model compression	(i) The use of convolutional layer factorization increases the number of kernel calls making each of them smaller	Achieva scanner (Philips Healthcare, Best, The Netherlands) with a pelvic phased-array coil (8 channel HD Torso XL)	90.9	3D	MRI	Prostate	Comelli et al.

V-Net [40]	(i) Fully CNN and suitable for volumetric medical image segmentation (ii) The residual function is learnt	(i) Location information is lost in the compression path	PROMISE 2012 Challenge	82.39	3D	MRI	Prostate	Milletary et al.

**Table 4:** Segmentation techniques: DeepLab V3, SegNet, and Fast Convolutional Network (FCN).

Method	Advantages	Disadvantages	Dataset	DC	ID	Modality	App	Ref
DeepLab V3 [41, 42]	(i) Allows us to enlarge the fields of view of filters to incorporate large context (ii) Preserves spatial information	(i) Has no postprocessing step conditional random fields (ii) Does not scale well for large or deeper layers if GPU memory is limited	CHAOS	81.0	3D	CT and MRI	Kidney	Guo et al.

SegNet [43]	(i) Low memory requirement during both training and testing (ii) Improved boundary delineation (iii) Reduced number of parameters enabling end to end training	(i) Both input image and output segmentation have fixed resolution	OASIS	91.47	3D	MRI	Brain	Khagi et al.

FCN [44, 45]	(i) Ability to make predictions on arbitrarily sized inputs (ii) End to end trainable fast and improved performance	(i) Direct predictions are typically in low resolution resulting in fuzzy object boundaries (ii) Suitable mainly for object detection, not object classification (used for local rather than global tasks)	DRIVE	95.33	3D	Funduscopy	Retinal vessels	Cai et al.

**(a):** 

Method	Description (texture features)	Advantage	Disadvantage
Gabor wavelet transform [52, 55, 58]	In information theory applications, Dennis Gabor used complex functions to build wavelets forming a basis for Fourier transforms.	Multiscale robust	Incomplete cover of spectrum plane needs rotation normalization
GLCM-based method [48]	Find the frequency of a set of pixel and its spatial relationship in an image to characterize its texture.	Easy to use compact robust	High computation cost partial description of texture

**(b):** 

Method	Description (colour features)	Advantage	Disadvantage
Scalable Colour Descriptor [48]	Defined in the hue-saturation-value (HSV) colour space with fixed colour space quantisation and uses a novel, Haar transform encoding	Compact and robust never changing and uninterrupted	Needs postprocessing for spatial information
Colour histogram [47, 48, 53]	A histogram represents the dispersion of colours in an image. It can be visualised as a graph that gives a high level of suspicion regarding the pixel value distribution	Simple to compute, easy to use and understand	High dimension sensitive to information

**(c):** 

Method	Description (shape features)	Advantage	Disadvantage
Wavelet transform [47]	Mathematical means for performing signal analysis when the signal frequency varies over time.	Translation and scale invariant good affine transformation good noise resistance	Average occultation resistance
Zernike moments [48]	A set of rotation invariant features is introduced. They are the magnitude of a set of orthogonal complex moments of the image.	Good noise resistance	High computational complexity bad affine transform

## Data Availability

No data has been used in this review research paper.
